# The Relationship between Thyroid-Stimulating Hormone and Insulin Resistance in Incipient Elderly Type 2 Diabetics with Normal Thyroid Function

**DOI:** 10.1155/2022/9447363

**Published:** 2022-03-07

**Authors:** Yajing Zhang, Lin Zhang

**Affiliations:** NHC Key Laboratory of Hormones and Development Tianjin Key Laboratory of Metabolic Diseases Chu Hsien-I Memorial Hospital & Tianjin Institute of Endocrinology, Tianjin Medical University, Tianjin 300134, China

## Abstract

**Objective:**

To explore correlations between serum thyroid-stimulating hormone (TSH) concentration within the normal range and insulin resistance and its possible mechanism in incipient type 2 diabetes in elderly patients.

**Methods:**

453 elderly patients with type 2 diabetes were divided into four groups by the quartile of TSH. Body mass index (BMI), waist-to-hip ratio (WHR), fasting plasma glucose (FPG), fasting insulin (FINS), homeostasis model assessment of insulin resistance (HOMA-IR) and homeostasis model assessment of insulin secretion (HOMA-*β*), blood lipids, and other indicators were compared among all groups, and correlation and regression analysis were conducted. 3T3-L1 preadipocytes were induced into mature adipocytes in vitro, and different concentrations of bovine TSH were used to stimulate adipocytes. The levels of TNF-*α* in the culture medium were detected by ELISA.

**Results:**

(1) With the increase of TSH, TC showed an increasing trend. Compared with the G1 group (4.80 ± 1.08), G2 group (5.13 ± 1.16), G3 group (5.14 ± 1.39), and G4 group (5.38 ± 1.16), the difference was statistically significant (*P* < 0.05 or *P* < 0.01). The LDL also showed an increasing trend. Compared with the G4 group (3.47 ± 0.89), the G1 (3.12 ± 0.82) and G2 groups (3.14 ± 1.05) had a lower LDL, and the difference was statistically significant (*P* < 0.01). The BMI increased between the G4 group (26.7 ± 3.97) and the G1 group (25.6 ± 3.54), and the difference was statistically significant (*P* < 0.05). (2) The serum TSH level was positively correlated with FPG, FINS, HOMA-IR, TC, and LDL (*R* = 0.292, 0.271, 0.394, 0.195, and 0.178, all *P* < 0.01). (3) TSH is the dependent variable, other indicators are independent variables, and multiple stepwise regression analysis is performed; the results show that only HOMA-IR, TC, and LDL enter the regression equation. (4) The TSH stimulated TNF-*α* secretion of 3T3-L1 adipocytes in a dose-dependent manner.

**Conclusion:**

The TSH level was positively correlated with the insulin resistance and LDL in the elderly incipient type 2 diabetic patients. Higher levels of TSH may be involved in the development of insulin resistance in the elderly incipient type 2 diabetic patients.

## 1. Introduction 

Type 2 diabetes mellitus (T2DM) is the most common type of diabetes in China, the majority of T2DM patients are middle-aged and elderly people, and the incidence is increasing year by year. Insulin resistance is the main pathophysiological basis of T2DM. In recent years, with the continuous in-depth research on the mechanism of insulin resistance, the role of thyroid-stimulating hormone (TSH) in the occurrence of insulin resistance has attracted much attention. The TSH binds to TSHR on the surface of adipocytes, then activates cyclic adenosine monophosphate-protein kinase A (cAMP-PKA) pathway, activates tumor necrosis factor-*α* (TNF-*α*) gene transcription and secretion of TNF-*α*, and further downregulates the expression of insulin receptor substrate-1 (IRS-1), which plays a role in insulin resistance. At present, under the premise of normal thyroid function, there are still few reports on the role of TSH in the onset of elderly type 2 diabetes patients. This study took newly-onset elderly type 2 diabetes patients as the research object and explored the correlation between serum TSH levels and insulin resistance and other metabolic indicators within the normal reference value range, in order to further understand the relationship between TSH and elderly type 2 diabetes and discuss its possible mechanism.

## 2. Method

### 2.1. Patients Test Indicators

From December 2018 to June 2020, 453 elderly patients with type 2 diabetes were enrolled in the study, who were first diagnosed during hospitalization in our hospital, aged 60 to 90 years old, with an average of 70.36 ± 7.19 years old. Among them, 236 were males and 217 were females. The diagnostic criteria for type 2 diabetes are in line with the 2013 American Diabetes Association (ADA). Diabetes is diagnosed by the following factors: fasting blood glucose ≥7.0 mmol/L and/or 2 h postprandial blood glucose ≥11.1 mmol/L [1]. None of the selected patients received any hypoglycemic drugs outside the hospital. Exclusion criteria for the patients include the following: patients with acute infection, diabetic hyperosmolar coma, diabetic ketoacidosis, acute and chronic heart failure, liver and kidney insufficiency, acute stroke patients, and patients with abnormal thyroid function during medication treatment.

Normal thyroid function is defined as TSH levels within 0.27–4.2 mIU/L, FT3 and FT4 are within the laboratory reference range (FT3 is 3.28–6.47 pmol/L and FT4 is 7.64–16.03 pmol/L). According to the patients' serum TSH levels, they were divided into four groups as follows: G1 group (TSH is 0.37–1.17 mIU/L), G2 group (TSH is 1.18–1.67 mIU/L), G3 group (TSH is 1.68–2.45 mIU/L), and G4 group (TSH 2.46–4.20 mIU/L). This study was approved by the Ethics committee of Zhu Xianyi Memorial Hospital, Tianjin Medical University. All patients signed the informed consent.

### 2.2. Detection of Indexes

Research subjects need to wake up in the morning, fasting, barefoot, and only wear underwear to measure height, weight, waist circumference, and hip circumference and calculate body mass index (BMI) and waist-hip ratio (WHR); at rest, the blood pressure (BP) was measured twice in the sitting position, and the average value was taken; fasting venous blood was taken, and biochemical indicators such as liver function, renal function, and blood lipid were measured by an automatic biochemical analyzer, and fasting plasma glucose (FPG) was determined by glucose oxidase method, and TSH, free triiodothyronine (FT3) and free thyroxine (FT4), fasting serum insulin (FINS), and glycosylated hemoglobin (HbA1c) were determined by chemiluminescence assay; using homeostasis model assessment for insulin resistance (HOMA-IR): HOMA-IR = FPG (mmol/L) × FINS (mIU/ml)/22.5 [2]. The homeostasis model was used to evaluate the insulin secretion index (HOMA-*β*): HOMA-*β* = 20 × FINS/(FPG-3.5) [3].

### 2.3. Culture and Induced Differentiation of 3T3-L1 Preadipocytes

The cells were inoculated in a cell culture flask at a cell density of 1.5 × 104/cm^2^, and the cells were placed in a high-sugar DMEM medium containing 10% calf serum at 37°C and 5% CO_2_ cell incubator for cultivation. The medium was changed every two days. When the cells grew to 60–70% confluence at the bottom of the culture flask in about 3-4 days, the cells were replaced with DMEM high glucose medium containing 0.5 mM IBMX, 1.0 M insulin, 0.25 M dexamethasone, and 10% FBS for 2 days (48 h). IBMX and dexamethasone were removed so that the complete medium contains only 1.0 M insulin. After 2 days, the medium was changed, and the insulin was removed. A complete medium is used without any inducer. The medium was changed every 2 days, and the differentiation was 8–10 days. Oil red O staining identification of induced differentiation 3T3-L1 cells was carried out.

### 2.4. Elisa Assay

After stimulation with different concentrations of bovine TSH (0.01 mIU/ml, 0.1 mIU/ml, and 1 mIU/ml) for 4 hours, the culture medium was collected strictly in accordance with the ELISA kit instructions. The enzyme-linked immunosorbent assay (ELISA) method was used to detect the concentration of TNF-*α* in the culture medium.

### 2.5. Statistical Methods

SPSS 20.0 software is used for statistical analysis. The data are represented by “”. Nonnormally distributed data are logarithmically transformed. Comparison between groups is performed by the analysis of variance. Pairwise comparison is performed by the LSD test. Correlation analysis is performed by the Pearson linear correlation analysis. Multivariate stepwise regression analysis was performed. The test level was *α* = 0.05. *P* < 0.05 indicated that the difference was statistically significant.

## 3. Results

### 3.1. Comparison of General Information of Patients

There were no significant differences in gender, age, systolic blood pressure, diastolic blood pressure, BMI, WHR, liver function, renal function, FT3, FT4, triglyceride (TG), and high-density lipoprotein (HDL) among 4 groups (*P* > 0.05). With the increase of TSH, the TC showed an increasing trend. Compared with the G1 group, G2 group, G3 group, and G4 group, the difference was statistically significant (*P* < 0.05 or *P* < 0.01). The LDL also showed an increasing trend. Compared with the G4 group, the G1, G2, and G3 groups, the difference was statistically significant (*P* < 0.01). As the TSH level increased, BMI of G1, G2, G3, and G4 groups also showed an upward trend, and the difference between the G4 and G1 groups was statistically significant (*P* < 0.05) (see Table 1).

### 3.2. Comparison of TSH Levels and Related Indicators of Glucose Metabolism in the Normal Range of Elderly Patients with Incient Type 2 Diabetes

There was no statistically significant difference in LnHOMA-*β* and HbA1c between groups of patients (*P* > 0.05). With the increase in serum TSH levels, FPG, FINS, and HOMA-IR all showed an upward trend. The pairwise comparison of G1, G2, and G3 groups showed no statistically significant difference (*P* > 0.05), while the comparison of the G4 group with G1, G2, and G3 groups showed statistically significant difference (*P* < 0.01), as shown in Table 2.

### 3.3. Correlation Analysis of Serum TSH Levels and Related Indicators

Correlation analysis of research subjects showed that serum TSH levels were positively correlated with FPG, FINS, HOMA-IR, TC, and LDL (*R* = 0.292, 0.271, 0.394, 0.195, and 0.178, all *P* < 0.01), and no correlation was found with HOMA-*β*, age, BMI, WHR, TG, HDL, SBP, DBP, and HbA1c, as shown in Table 3.

### 3.4. Multiple Stepwise Regression Analysis

Using TSH as the dependent variable, using FPG, FINS, HOMA-IR, TC, and LDL as independent variables, multiple stepwise regression analysis was performed. The results showed that HOMA-IR, TC, and LDL entered the regression equation; HOMA-IR, TC, and LDL were independently correlated with TSH. The regression equation was as follows: *Y* = 0.393 + 0.187*X*1 + 0.103*X*2 + 0.092*X*3 (*X*1: HOMA-IR; *X*2: TC; X3: LDL; *P* < 0.05).

### 3.5. Culture and Induced Differentiation of 3T3-L1 Preadipocytes

The morphology of mouse 3T3-L1 preadipocytes and fibroblasts is similar, as shown in Figures 1(a) and 1(b). After induction to the 10th day, lipid droplets of varying sizes were seen in most of the cells, and the cell volume increased to fill the intercellular space. After oil red O staining, there are bright red particles in the cytoplasm of induced differentiated mature adipocytes. After hematoxylin counterstaining, the nucleus was blue and deviated from the center of the cell. Observed under a 10x light microscope, randomly counted the proportion of adipocytes in the total number of cells in 10 nonrepetitive fields, and more than 95% showed adipocyte phenotype, which was further confirmed to be mature adipocytes.

### 3.6. Effect of TSH on the Secretion of TNF-*α* in 3T3-L1 Adipocytes

The 3T3-L1 adipocytes were stimulated with different concentrations of bovine TSH to induce differentiation and mature 3T3-L1 adipocytes for 4 hours, and the TNF-*α* level in the culture medium was detected. The results showed that, with the increase of TSH stimulation concentration, the TNF-*α* level showed an upward trend, and the difference was statistically significant as shown in Figure 1(c).

## 4. Discussion

Insulin resistance is an important pathophysiological basis for the occurrence of T2DM. The previous research centers on the pathogenesis of diabetes, most of the focus was on the secretion of inflammatory factors from adipocytes to cause insulin resistance, and then diabetes, ignoring that factors other than inflammatory factors would also participate in the occurrence of insulin resistance and metabolic disorders. In the past, thyroid disease was considered to be an endocrine metabolic disease independent of diabetes. In recent years, the relationship between TSH and diabetes and diabetic ischemic heart disease has gradually attracted attention. A large number of studies have shown that [4–6], diabetic patients, especially combined among diabetic patients with cardiovascular disease, the prevalence of abnormal thyroid function is significantly higher than that of nondiabetic patients.

In recent years, research on TSH levels and insulin resistance in people with normal thyroid function has gradually attracted attention. A study by Roos et al. on 2703 patients without thyroid disease and diabetes showed that serum TSH levels were significantly positively correlated with HOMA-IR [7]. Jayanthi R et al. found that serum TSH levels were positively correlated with plasma insulin level and significantly negatively correlated with the insulin sensitivity index with 530 normal, overweight, and obese adults [8]. Similarly, we also found in the previous study that the serum TSH level of T2DM patients was significantly higher than that of the normal control group [9]. In our previous study on diabetic rats, we found that the serum TSH level was negatively correlated with the insulin sensitivity index [10]. Preliminary research suggests that the TSH may be involved in the occurrence of insulin resistance and further development of type 2 diabetes. At present, the correlation between TSH and insulin resistance in elderly T2DM patients is still rarely reported. This study took newly onset elderly patients with type 2 diabetes as the research object, explored the correlation between serum TSH and insulin resistance and related metabolic indicators within the normal reference value range, and explored whether TSH is associated with the occurrence of newly onset elderly T2DM insulin resistance and abnormal lipid metabolism so as to provide a basis for further clinical treatment.

The results of this study suggest that, with the increase in serum TSH levels, BMI, TC, LDL, FINS, and HOMA-IR all showed an upward trend, while HOMA-*β* showed a downward trend, the TSH was within the normal range, and FNS and HOMA-IR are positively correlated in newly onset elderly patients with type 2 diabetes. Further cytological studies have shown that the TSH can stimulate 3T3-L1 adipocytes to secrete TNF-*α* in a dose-dependent manner (*P* < 0.05) and TSH can increase the activity of NF-кB. As can be seen from the gel electrophoresis pattern, the NF-кB/DNA probe binding bands gradually increased with the increase of TSH stimulation concentration. This effect was inhibited by a PKA inhibitor (H89). The possible mechanism is analyzed as follows: (1) our previous research results confirmed that there is the expression of thyroid-stimulating hormone receptor (TSHR) on the surface of adipocytes, TSH binds to TSHR on the surface of adipocytes, then activates the cyclic adenosine monophosphate-protein kinase A (cAMP-PKA) pathway [11–13], activates tumor necrosis factor-*α* (TNF-*α*) gene transcription and secretion of TNF-*α*, further downregulates the expression of insulin receptor substrate-1 (IRS-1), and interferes with the normal tyrosine phosphorylation of IRS-1, which plays a role in insulin resistance; (2) insulin resistance can lead to a compensatory increase in early insulin levels, and insulin increases TSH levels by affecting the level of leptin [14]; (3) overweight and obesity are one of the important causes of insulin resistance. This study found that, with the increase of TSH level, the BMI of patients showed an increasing trend, and the difference between the G4 group and the G1 group was statistically significant (*P* < 0.05). The reason may be that obesity leads to leptin resistance, resulting in serum leptin excess, which upregulates the expression of thyrotropin-releasing hormone and further increases serum TSH level [15, 16]. All of these mechanisms can lead to elevated TSH to further aggravate the occurrence of insulin resistance.

This study further found that the TSH is positively correlated with TC and LDL in the normal range. This may be because TSH directly acts on TSHR on liver cell membranes and stimulate cyclic adenosine mono-acyl-CoA reductase, and it also promotes cholesterol synthesis through the cyclic adenosine monophosphate/protein kinase A/cyclic adenosine phosphate response element-binding protein (cAMP/PKA/CREB) signaling system [17, 18]. Abnormal blood lipid metabolism may further damage the body's defense against oxidative stress, cause damage to the function of vascular endothelial cells and accelerate the formation of atherosclerosis, and increase the risk of cardiovascular disease.

To sum up, in the newly onset elderly type 2 diabetes patients with normal thyroid function, serum TSH levels are positively correlated with TC and LDL, and higher TSH levels within the normal reference value range may play a promoting role in the occurrence and development of insulin resistance through the abovementioned mechanisms. The elevated TC and LDL further participate in the pathological process of atherosclerosis occurs and increase the risk of cardiovascular disease in elderly patients with type 2 diabetes.

Therefore, it is necessary to strengthen thyroid function in elderly patients with type 2 diabetes. Monitoring and timely attention to the risk factors related to cardiovascular disease in patients with normal thyroid function and high serum TSH levels will play a positive role in preventing and delaying the occurrence of cardiovascular complications in elderly patients with type 2 diabetes.

Therefore, monitoring of thyroid function in elderly patients with type 2 diabetes should be strengthened, and timely attention should be paid to the risk factors related to cardiovascular disease in patients with normal thyroid function and high serum TSH levels, which will play a positive role in preventing and delaying the occurrence of cardiovascular disease in elderly patients with type 2 diabetes.

## Figures and Tables

**Figure 1:** Culture and induced differentiation of 3T3-L1 preadipocytes. (a) 3T3-L1 preadipocytes (×100). (b) 3T3-L1 adipocytes (×100). (c) Different concentrations of TSH stimulated the level of TNF-*α* in the culture medium of 3T3-L1 adipocytes. ^*∗*^*P* < 0.05 and ^*∗∗*^*P* < 0.01.

**Table 1:** Comparison of clinical characteristics of different TSH patients.

Group	G1 (TSH 0.37–1.17 mIU/L)	G2 (TSH 1.18–1.67 mIU/L)	G3 (TSH 1.68–2.45 mIU/L)	G4 (TSH 2.46–4.20 mIU/L)
N ((F/M))	113 (51/62)	113 (52/61)	113 (59/54)	114 (56/58)
Age (year)	70.0 ± 7.09	70.6 ± 6.98	70.8 ± 8.08	70.1 ± 6.58
WHR (g/cm^2^)	0.91 ± 0.08	0.92 ± 0.07	0.93 ± 0.07	0.91 ± 0.08
BMI (kg/m^2^)	25.6 ± 3.54	25.8 ± 3.63	26.5 ± 3.57	26.7 ± 3.97^a^
SBP (mmHg)	127 ± 15.7	127 ± 14.1	129 ± 14.0	126 ± 13.8
DBP (mmHg)	77.6 ± 9.69	75.6 ± 10.5	77.5 ± 9.91	77.0 ± 8.92
TG (mmol/L)	1.90 ± 1.33	2.14 ± 1.54	2.10 ± 1.24	2.08 ± 1.33
TC (mmol/L)	4.80 ± 1.08	5.13 ± 1.16^a^	5.14 ± 1.39^a^	5.38 ± 1.16^b^
LDL (mmol/L)	3.12 ± 0.82	3.14 ± 1.05	3.27 ± 0.90	3.47 ± 0.89^bd^
HDL (mmol/L)	1.33 ± 0.42	1.25 ± 0.29	1.26 ± 0.32	1.25 ± 0.28
FT_3_ (pmol/L)	10.8 ± 6.25	10.1 ± 6.54	10.2 ± 6.50	9.53 ± 5.41
FT_4_ (pmol/L)	12.1 ± 6.09	12.0 ± 6.67	11.6 ± 6.65	12.6 ± 5.67
ALP (U/L)	69.5 ± 15.7	71.4 ± 18.4	71.9 ± 19.6	73.3 ± 18.8
GGT (U/L)	35.2 ± 20.9	33.6 ± 20.9	32.8 ± 20.4	32.3 ± 18.8
ALT (U/L)	29.6 ± 18.6	26.3 ± 15.1	26.5 ± 16.6	27.3 ± 17.5
AST (U/L)	23.1 ± 13.3	20.8 ± 9.31	22.6 ± 13.8	20.9 ± 9.52
BUN (mmol/L)	5.60 ± 1.30	5.44 ± 1.32	5.45 ± 1.36	5.45 ± 1.64
Cre (umol/L)	67.2 ± 14.6	63.8 ± 15.4	64.3 ± 14.5	66.1 ± 20.6
UA (umol/L)	307 ± 96.5	305 ± 87.9	314 ± 92.5	312 ± 93.5

*Note.* Compared with G1, ^a^*P* < 0.05, ^b^*P* < 0.01; compared with G2, ^c^*P* < 0.05, ^d^*P* < 0.01; and compared with G3, ^e^*P* < 0.01.

**Table 2:** Comparison of related indicators of glucose metabolism in different TSH patients.

Group	G1 TSH 0.37–1.17 mIU/L	G2 TSH 1.18–1.67 mIU/L	G3 TSH 1.68–2.45 mIU/L	G4 TSH 2.46–4.20 mIU/L
N ((F/M))	113 (51/62)	113 (52/61)	113 (59/54)	114 (56/58)
FPG (mmol/L)	8.42 ± 2.31	8.20 ± 2.24	8.37 ± 1.96	10.4 ± 3.09^bde^
FINS (mIU/L)	9.03 ± 3.18	9.15 ± 5.02	9.24 ± 4.05	11.8 ± 4.27^bde^
HOMA-IR	3.34 ± 1.39	3.30 ± 2.03	3.42 ± 1.71	5.37 ± 2.46^bde^
LnHOMA-*β*	3.65 ± 0.66	3.63 ± 0.80	3.61 ± 0.71	3.57 ± 0.61
HbA_1_c	8.76 ± 2.05	9.02 ± 2.11	8.90 ± 1.97	8.70 ± 1.95

*Note.* Compared with G1, ^a^*P* < 0.05 and ^b^*P* < 0.01; compared with G2, ^c^*P* < 0.05 and ^d^*P* < 0.01; and compared with G3, ^e^*P* < 0.01.

**Table 3:** Correlation analysis of serum TSH level.

Statistics	FPG	FINS	HOMA-IR	TC	LDL
*r*	0.292	0.271	0.394	0.195	0.178
*P*	<0.001	<0.001	<0.001	<0.001	<0.001

## Data Availability

The data used to support the findings of this study are available on reasonable request from the corresponding author.
